# Effects of curcumin on glycemic control and lipid profile in prediabetes and type 2 diabetes mellitus: A systematic review and meta-analysis

This article has been retracted.

**DOI:** 10.1371/journal.pone.0215840

**Published:** 2019-04-23

**Authors:** Nalinee Poolsup, Naeti Suksomboon, Putu Dian Marani Kurnianta, Kulchalee Deawjaroen

**Affiliations:** 1 Department of Pharmacy, Faculty of Pharmacy, Silpakorn University, Nakhon-Pathom, Thailand; 2 Department of Pharmacy, Faculty of Pharmacy, Mahidol University, Bangkok, Thailand; Weill Cornell Medical College Qatar, QATAR

## Abstract

**Scope:**

Studies have demonstrated inconsistent effects of curcumin on glycemic outcomes and lipid parameters in patients with prediabetes and type 2 diabetes mellitus (T2DM). This study aimed to assess the effect of curcumin on glycemic control and lipid profile in prediabetes and T2DM.

**Methods and results:**

A systematic search of randomized controlled trials (RCTs) was conducted from inception to June 2018 in electronic sources including AMED, ANZCTR, BioMed Central, CENTRAL, CINAHL, ClinicalTrials.gov, Expanded Academic Index, Google Scholar, ISRCTN, LILACS, MEDLINE, NCCIH, Science Direct, Scopus, Web of Science, and WHO ICTRP. Hand search was also performed. Of the total 486 records, four trials (N = 508) and eight trials (N = 646) were eligible for the meta-analysis of individuals with prediabetes and T2DM, respectively. Curcumin significantly reduced glycosylated hemoglobin (HbA1c) in prediabetics (MD: -0.9%, 95% CI: -1.7 to -0.1%, p = 0.03). Furthermore, T2DM subjects gained favorable reduction in both HbA1c (MD: -0.5%, 95% CI: -1.0 to -0.0%, p = 0.04) and fasting plasma glucose (MD: -11.7 mg/dL, 95% CI: -22.1 to -1.3 mg/dL, p = 0.03). Tendency of lipid profile improvement was also observed.

**Conclusion:**

Our findings may encourage curcumin supplementation based on its meaningful effect on glycemic control and positive trend on lipid outcomes in prediabetes and T2DM.

## Introduction

Diabetes is a metabolic disease presenting with elevated blood glucose level. This disease accounted for not only 1.5 million deaths in 2012, but also an extra 2.2 million deaths for its attribution to cardiovascular disease and other diseases. Accordingly, diabetes has become a worldwide burden especially in less developed countries [1]. Furthermore, the global prevalence of diabetes has been predicted to keep increasing to 13.5% of the total world population in 2040 [2]. Among the growing number of people with diabetes, type 2 diabetes mellitus (T2DM) is the most prevalent. In order to manage with the worldwide issues of diabetes, effective prevention and management are entirely required.

T2DM is preventable disorder [1]. Prevention should also be initiated in people with prediabetes or impaired glucose tolerance who are prone to T2DM. Lifestyle modification and pharmacologic intervention are suggested [3]. However, single oral antidiabetic drug may poorly control blood glucose at times. Consequently, additional insulin seems to take some cost and patient preference issues. This may grow another problem as the economic burden of diabetes treatment has affected many countries around the world [4]. Hence, the more affordable alternative therapy for diabetes, either as additional supplement or as prevention is necessary. Herbal medicine is an interesting approach for diabetes treatment. Some evidence has conclusively demonstrated the efficacy of medicinal plants in prediabetes and type 2 diabetes mellitus [5, 6].

Curcumin is an active ingredient contained in the rhizome of *Curcuma longa* plant or turmeric. This natural substance has purported anti-inflammatory, anti-depressant, and anti-diabetic effects [7]. Animal study revealed that curcumin and its analogues resembled the action of antidiabetic drug namely thiazolidinedione group through activation of peroxisome proliferator-activated receptor-γ (PPAR-γ) [8]. Thus, curcumin may correct the responsible targets relating to glucose and lipid control in the body [9] which play an important part in diabetes management [3]. Curcumin’s effects on glycemic outcomes and lipid parameters have been translated in human through several randomized controlled trials enrolling subjects with prediabetes [10, 11] and T2DM [12–14]. The inconsistency among the results of those studies has raised a question regarding the role of curcumin in diabetes management. Therefore, we performed this systematic review and meta-analysis to assess the effect of curcumin on glycemic control and lipid profile in prediabetes and T2DM.

## Materials and methods

We conducted a systematic review and meta-analysis according to the Preferred Reporting Items for Systematic Reviews and Meta-analysis (PRISMA) guidelines [15].

### Search strategy and study selection

We carried out a systematic search through bibliographic databases or search engines including Allied and Complementary Medicine Database (AMED), BioMed Central, Cochrane Central Register of Controlled Trials (CENTRAL), Cumulative Index to Nursing and Allied Health Literature (CINAHL), Dissertation Abstracts International (DAI), ProQuest Dissertations and Theses (PQDT), Expanded Academic Index, Google Scholar, Latin American and Caribbean Health Sciences Literature (LILACS), MEDLINE (Pubmed), National Center for Complementary and Integrative Health (NCCIH), Science Direct, Scopus, and Web of Science. We also searched clinical trial registry databases including Australian New Zealand Clinical Trials Registry (ANZCTR), ClinicalTrials.gov, World Health Organization International Clinical Trial Registry Platform (WHO ICTRP), and International Standard Randomized Controlled Trial Number (ISRCTN). MeSH terms were used to include diabetes mellitus, prediabetic state, curcumin, curcuma, hypoglycemic agents, placebos, blood glucose, glycated hemoglobin A, triglycerides, (cholesterol, HDL), (cholesterol, LDL), insulin resistance, hyperglycemia. We applied the following keywords: curcum*, curcumin extract, curcuma extract, turmeric, turmeric extract, curcuminoid(s), HbA1c, lipid, lipid profile(s), prediabetes, antidiabetic, and type 2 diabetes. The search strings were combined by using Boolean operators. Additionally, hand search was performed to find relevant cited articles from reference list of the identified articles. We conducted all the searches from respective inceptions until the end of June 2018.

We included the studies if they met the following criteria: (i) randomized controlled trials (RCTs) comparing the effect of curcumin preparation or turmeric powder to placebo; (ii) involved participants with prediabetes or type 2 diabetes mellitus (T2DM); (iii) reported glycemic parameters used in clinical practice such as, glycosylated hemoglobin (HbA1c) or fasting plasma glucose (FPG) [3] with or without the report of lipid outcomes including total cholesterol (TC), triglycerides (TG), HDL, or LDL; and (iv) treatment duration of at least 8 weeks. Eight-week duration was considered sufficient to obtain meaningful effect since we decided HbA1c as our primary outcome [16]. FPG and lipid profile were determined as secondary outcomes. We did not restrict the publication language, so we had the non-English articles translated into English. We independently screened the records based on their titles and abstracts. PDMK further reviewed and selected the obtained full-text articles according to the inclusion criteria. NS and NP finalized the eligibility for meta-analysis.

### Data extraction and quality assessment

Two reviewers (PDMK, NP) independently extracted the data for meta-analysis, evaluated the quality of qualified studies, and performed double-check. NS resolved the disagreements, if necessary. The following data were extracted in standardized form: (i) studies’ characteristics, including authors, year, design, location, duration, and intervention arms; (ii) subjects’ information, including inclusion criteria, age, and gender; (iii) outcomes assessed, including baseline and endpoint values of main outcomes of interest (HbA1c, FPG, TG, TC, LDL, and HDL). The outcomes values were managed in the same unit for HbA1c (%), FPG (mg/dL), and lipid profile (mg/dL). If we found the other treatment arms than curcumin and placebo, we only extracted the data from curcumin and placebo groups for prediabetes or T2DM studies. The studies’ quality was evaluated using Cochrane Risk of Bias Tool [17]. We considered the methodological domains of individual studies as low risk, high risk, or unclear risk of bias. The seven domains in the assessment involved random sequence generation, allocation concealment, blinding of participants and personnel, blinding of outcome assessment, incomplete outcome data, selective outcome reporting, and other risk of bias.

### Statistical analysis

Meta-analysis was performed for prediabetes and T2DM using Review Manager Software (RevMan version 5.3.5). We estimated the treatment effects on HbA1c, FPG, TC, TG, LDL, and HDL by pooling mean and SD of endpoint values in the treatment and control groups. Final values were decided for these data based on assumption of similar direction given by the effect magnitude. In the absence of both data, we converted the available statistical data into mean and SD by applying appropriate formula [17, 18]: Mean = median; SD = range/6 (when n > 70); SD = SEM × √n (values within group); or SD = IQR/1.35 (symmetrical data distribution), where SD is the standard deviation, n is group size, SEM is standard error of the mean, and IQR is interquartile range, consecutively. The pooled data were computed using inverse variance-weighted method and presented as weighted mean difference (MD) with 95% CI. The degree of heterogeneity was defined based on I-squared statistic. The heterogeneity was substantially significant when the Cochrane’s test showed I^2^ greater than 50% with p-value <0.1. Data with significant heterogeneity were analyzed using DerSimonian and Laird random-effect model, otherwise, a fixed-effect model was applied. The results of meta-analysis were statistically significant at the level of 0.05 based on Z-score of overall effects [17, 19]. Sensitivity analysis was undertaken to observe if curcumin is effective for the treatment with short duration according to the duration criteria in this systematic review. Publication bias was evaluated based on funnel plot and Egger’s regression test [20].

## Results

### Summary of selected studies

Fig 1 represents the search process. We retrieved a total of 486 records from the electronic sources and manual search. There were 35 full-texts of RCTs qualified for further eligibility assessment following title and abstract screening. Among these articles, we excluded 23 trials by the following reasons: four were conducted in other populations [21–24]; nine trials tested curcumin as combination [25–33]; two trials were not controlled trials [34, 35]; six trials did not provide our outcomes of interest [36–41]; and the rest two trials were less than 8 weeks duration [42, 43]. Hence, we finally included 12 studies [10–14, 44–50] for the systematic review and meta-analysis. Of these, there were 2 non-English articles which were translated into English [12, 50].

**Fig 1:** PRISMA flow diagram of the study selection.

### Studies’ characteristics and risk of bias

The summary of the main features of the included studies is shown in Table 1. We obtained four trials in prediabetes involving 508 participants in Asian countries [10, 11, 44, 45]. These participants seemed to have similar characteristics. However, one study [45] recruited only male subjects. All studies in prediabetes, except one add-on study [10], tested curcumin as single supplementation. Adverse events (AEs) were assessed in all prediabetes studies along with outcomes of interest and the other varied outcomes. The remaining eight studies were conducted in 646 subjects with T2DM [12–14, 46–50]. All of these studies were performed in Asian countries, except one study [48] in Mexico. The background characteristics of subjects with T2DM were more varied than those of subjects with prediabetes. These attributes were for example, diabetic nephropathy, chronic kidney disease, and suspected coronary artery disease. All studies in T2DM were add-on trials, except two studies [14, 48]. One study was conducted in Naïve T2DM participants and tested curcumin without background therapy [14]. A study did not clearly mention the background medication [48]. Only 3 studies in T2DM assessed AEs. The preparation forms of curcumin studied in all trials of both prediabetes and T2DM included curcuminoid extract 300 mg to 1.8 g per day, turmeric powder 1.5 g to 2.4 g per day, curcumin amorphous dispersion 500 mg per day, standardized curcuminoids preparation 600 mg per day, and nano-curcumin 80 mg per day.

**Table 1:** Characteristics of included studies and participants.

Study	Design (location, duration)	N	Inclusion criteria	Study arms and participants (size, mean age ± SD)	Co-treatment	Outcomes findings^a^	Other assessed outcomes
**Prediabetes**							
Chuengsamarn et al. (2012) [44]	RP, DB (Thailand, 9 months)	237	Naïve prediabetes (American Diabetes Association criteria), age ≥ 35 years	T: Curcumin capsule (curcuminoids extract 1.5 g/day); F/M: 78/42; age: 57.0 ± 12.1 years C: Placebo; F/M: 75/42; age: 58.9 ± 12.8 years	Healthy lifestyle education, no medication	HbA1c↓, FPG↓, 2HPP↓, minor AEs (T/C: 4/0)	β-cell functions, insulin resistance, obesity, BMD, liver enzymes, creatinine, anti-inflammatory cytokine
Yang et al. (2014) [10]	RP, DB (Taiwan, 12 weeks)	65	MetS (prediabetes, prehypertension, DLP), Asian populations	T: Curcumin capsule (curcuminoids extract 95% 1.9 g/day = 1.8 g/day); F/M: 21/12; age: 59.0 ± 10.1 years C: Placebo; F/M: 15/17; age: 59.6 ± 14.1 years	Stable treatment (started at least 6 months before study)	HbA1c↓, FPG↔, TG↔, TC↔, LDL↔, HDL↑, AEs (T/C: 3/0)	Anthropometrics^b^, other metabolic parameters (VLDL, non-HDL, TC/HDL ratio)
Amin et al. (2015) [45]	RP, DB (Pakistan, 8 weeks)	126	MetS (prediabetes, prehypertension, DLP), male resident of Hijrat colony	T: Turmeric powder in capsule 2.4 g/day; M: 63; age: 42.4 ± 13.7 years C: Placebo; M: 63; age: 41.6 ± 12.8 years Others: Black seeds and combination	Healthy lifestyle education, no medication	FPG↔, TG↔, TC↔, LDL↓, HDL↑, AEs (T/C: 4/0)	Anthropometrics^b^, BP, c-reactive protein
Rahmani et al. (2016) [11]	RP, DB (Iran, 8 weeks)	80	MetS (prediabetes, prehypertension, DLP), NAFLD (grades 1–3)	T: Curcumin capsule (curcumin amorphous dispersion 500 mg/day = curcuminoids 70 mg/day); F/M: 19/21; age: 46.4 ± 11.6 years C: Placebo; F/M: 19/21; age: 49.0 ± 9.8 years	No medication	HbA1c↓, FPG↓, TG↔, TC↓, LDL↓, HDL↑, no severe AEs (T/C: 3/0)	Anthropometrics^b^, liver enzymes, NAFLD severity (liver ultrasonography)
**Type 2 Diabetes Mellitus**							
Usharani et al. (2008) [46]	RP (India, 8 weeks)	44	T2DM, age 21–80 years, on stable antidiabetic agents ≥2 months	T: NCB-02 (standardized C3 curcuminoids preparation) 600 mg/day; F/M: 11/12, age: 55.5 ± 10.7 years C: Placebo; F/M: 10/11, age: 49.8 ± 8.2 years Other: Atorvastatin	Metformin or metformin + sulfonylurea	HbA1c↔, FPG↔, TG↔, TC↓, LDL↔, HDL↔, no serious AEs (T/C: 2/0)	Endothelial function, biomarker levels (endothelin-1, tumor necrosis factor-α, interleukin-6, malondialdehyde)
Khajehdehi et al. (2011) [47]	RP, DB (Iran, 2 months)	40	Overt type 2 diabetic nephropathy (poorly controlled), proteinuria ≥ 500 mg/day, normal kidney function, well-controlled BP	T: Turmeric powder in capsule 1.5 g/day = curcumin 66.3 mg/day; F/M: 11/9; age: 52.9 ± 9.2 years C: Placebo; F/M = 7/13, age: 52.6 ± 9.7 years	Usual lifestyle, stable ACEI and/ or ARB (no detail of specific agent)	FPG↔, 2HPP↔, TG↔, TC↔, LDL↔, HDL↔, no case of AEs reported (T/C: 0/0)	interleukin-8, and tumor necrosis factor- α
Adab et al. (2013) [12]	RP, DB (Iran, 8 weeks)	75	Hyperlipidemic non-insulin T2DM, age 30–70 years, not taking supplement in the last 3 months, BMI 20.0–35.0 kg/m^2^	T: Turmeric powder in capsule 2.1 g/day; F/M: 20/19: age: 54.7 ± 6.0 years C: Placebo; F/M: 19/17: age: 55.7 ± 8.6 years	Stable lifestyle, OAD (metformin, glibenclamide, gliclazide or combined), LLD (atorvastatin cholestyramine, fenofibrate, or gemfibrozil)	HbA1c↓, FPG↓, TG↓, TC↔, LDL↓, HDL↔, AEs not assessed	Insulin resistance, apolipoprotein A-1 and B, physical activity frequency
Na et al. (2013) [13]	RP, DB (China, 3 months)	100	Overweight or obese T2DM, age 18–65 years, BMI ≥24.0, on optimal treatment ≥ 6 months	T: Curcuminoids capsule (curcuminoids 300 mg/day); F/M: 26/24; age: 55.4 ± 6.4 years Placebo; F/M: 25/25; age: 54.7 ± 8.3	Usual lifestyle, OAD or insulin or both + LLD or AHT (ACEI or ARB or ACEI + ARB or other AHT)	HbA1c↓, FPG↔, TG↔, TC↔, LDL↔, HDL↔, AEs not assessed	Anthropometrics^b^, BP, dietary intake, insulin resistance, hematology, apolipoprotein A-1 and B, liver enzyme markers
Chuengsamarn et al. 2014 [14]	RP, DB (Thailand, 6 months)	213	Naïve T2DM (American Diabetes Association criteria), age ≥35 years	T: Curcumin capsule (curcuminoids extract 1.5 g/day); F/M: 57/50; age: 59.2 ± 11.0 years C: Placebo; F/M: 59/47; age: 59.6 ± 10.7 years	Healthy lifestyle education, no medication	HbA1c↓, FPG↓, TG↔, TC↓, LDL↓, HDL↑, minor AEs (T/C: 4/4)	Average pulse wave velocity, uric acid, adipocytokines, insulin resistance, abdominal obesity, creatinine, liver enzymes
Jiménez-Osorio et al. 2016 [48]	RP, DB (Mexico, 8 weeks)	51	Diabetic and nondiabetic proteinuric chronic kidney disease without urinary tract infection or heart failure (class III or IV), age 20–70 years, Mexican population	T: Turmeric capsule (curcumin 320 mg/day); F/M: 9/19 age: 55.0 ± 8.5 years C: Placebo; F/M: 6/17; age: 56.2 ± 7.2 years	Usual lifestyle, no information of medication	FPG↓, TG↔, TC↔, AEs not assessed	Anthropometrics^b^, BP, protein urea, oxidative stress markers, antioxidant capacity, activity of antioxidant enzymes, nuclear factor erythroid-2 related factor activity
Rahimi et al. 2016 [49]	RP, DB (Iran, 3 months)	70	Suspected coronary artery disease, male or female age >18 years, T2DM	T: Nano-curcumin (nano-micelle) 80 mg/day; F/M: 18/17; age: 56.3 ± 11.2 years C: Placebo; F/M: 21/14, age: 70.0 ± 10.8 years	Healthy lifestyle education, necessary medications (no detail provided)	HbA1c↓, FPG↓, estimated average glucose↓, TG↑, TC↔, LDL↔, HDL↑, AEs not assessed	Body mass index
Hodaie et al. 2017 [50]	RP, DB (Iran, 10 weeks)	53	T2DM diagnosed for 1–10 year, without insulin, age 40–70 years, BMI 18.5–30.0 kg/m2	T: Curcumin capsule 1.5 g/day = curcuminoids 1.3 g/day; F/M: 10/15; age: 57.0 ± 8.0 years C: Placebo; F/M: 18/10; age: 60.0 ± 7.0 years	Usual lifestyle, medication: OAD (Met, Glibenclamide, Met + Gli, others), LLD, AHT (half user)	HbA1c↔, FPG↓, AEs assessment not clearly defined	Anthropometrics^b^, dietary intake, insulin resistance, insulin

ACEI, angiotensin converting enzyme inhibitors; AEs, adverse events; AHT, antihypertension; BMD, bone mineral density; BP, blood pressure; DB, double-blinding; DLP, dyslipidemia; F/M, female/male; LLD, lipid lowering drugs; MetS, metabolic syndrome; NAFLD, non-alcoholic fatty liver disease; OAD, oral antidiabetic drugs; RP, randomized parallel design; T2DM, type 2 diabetes mellitus; T/C, treatment/control; 2HPP, 2-hours postprandial glucose

^a^Arrows represent relative comparison of change from baseline between treatment group and control group (opposite direction or similar direction with control group).

^b^Anthropometric assessments were varied such as body weight, body mass index, waist circumference, or hip circumference.

All trials were randomized trials, but half number of studies did not appropriately describe the method of randomization and allocation concealment. Consequently, the risk of selection bias remained unclear across those studies. All studies demonstrated low risk of performance bias by performing double-blinded method. However, one study [46] did not specify the blinding method. We considered this study as having high risk of performance bias since we found its interventions were distinguishable. These interventions probably affect the outcome assessment, therefore we judged the risk of detection bias of the referred study as high. Meanwhile, majority of the other studies had unclear risk in detection bias. There was no remarkable attrition bias, reporting bias, and other bias across studies. Nevertheless, one study [45] revealed high risk of attrition bias. Two studies had high risk in reporting bias [46, 50] and one study likely showed high risk of other bias due to imbalance baseline values [11], respectively. The risk of bias evaluation is provided in Fig 2 and S1 Fig.

**Fig 2:** Risk of bias summary for each included study. (+) low risk of bias, (-) high risk of bias, (?) unclear risk of bias.

### Meta-analysis on glycemic control and lipid profile in prediabetes

Random-effect model was performed in pooling the data on glycemic outcomes in prediabetes due to the significantly high heterogeneity (I^2^ = 92%, p<0.00001). Four studies [10, 11, 44, 45] in prediabetes with 496 subjects contributed for the meta-analysis on FPG. However, one study [45] did not provide HbA1c leaving the analysis on this outcome with only three studies of 370 subjects. The results revealed that the mean differences between curcumin and placebo groups were -0.89% (95% CI: -1.70 to -0.08%, p = 0.03) on HbA1c and -10.77 mg/dL (95% CI: -22.65 to 1.12 mg/dL, p = 0.08) on FPG, respectively. These findings indicated the significant effect of curcumin in reducing HbA1c in prediabetes (Fig 3).

**Fig 3:** Meta-analysis of glycemic outcomes in prediabetes and type 2 diabetes mellitus.

The meta-analysis on all lipid outcomes in prediabetes consisted of three studies [10, 11, 45] with 262 participants. Positive effects on lipid outcomes were explained as a decrease in TG, TC, and LDL, but an increase in HDL. Regardless of the varied heterogeneity (I^2^ = 0–92%) and analysis model, curcumin demonstrated non-significant effects on lipid profile (S2 Fig).

Sensitivity analysis regarding the duration of the treatment by removing study with far longer duration [44] was planned. However, due to the limited number of studies after removal, we did not proceed with the analysis.

### Meta-analysis on glycemic control and lipid profile in T2DM

The data of glycemic outcomes in T2DM demonstrated significant heterogeneity (I^2^ = 68–72%, p = 0.003). Based on the meta-analysis of six trials (N = 546) [12–14, 46, 49, 50], curcumin offered benefit of HbA1c reduction by up to -0.49% (95% CI: -0.96 to -0.02%, p = 0.04). Consistently, the result on FPG from eight trials (N = 637) [12–14, 46–50] offered favorable lowering effect (MD: -11.68 mg/dL, 95% CI: -22.11 to -1.25 mg/dL, p = 0.03). Therefore, curcumin contributed to significant improvement on glycemic control in T2DM (Fig 3).

Significant heterogeneity was also found in the meta-analysis on lipid outcomes in T2DM (I^2^ = 71–89%, p≤0.002). Random effect model was applied to pool the data in both TG and TC involving seven trials (N = 593) [12–14, 46–49]. By removing one study [48] which did not provide outcomes on LDL and HDL, we performed the analysis for the remaining six trials (N = 542) under the same model. Curcumin seemed to have greater effect in lipid outcomes including TG, TC, and HDL toward T2DM population than prediabetes population. Nevertheless, the overall effect on all lipid outcomes in T2DM again did not indicate significant results (S3 Fig).

We undertook sensitivity analysis in T2DM by removing one studies conducted in much longer duration [14] than the majority of the studies. We summarized the results of sensitivity analysis on glycemic outcomes and lipid outcomes in S1 Table. The results on glycemic parameters were affected to become non-significant. Meanwhile, the results on lipid outcomes did not change regardless of the treatment duration.

### Publication bias

We tested the risk of publication bias by funnel plot and Egger’s regression test in the presence of at least five studies. We planned to evaluate the publication bias of studies in prediabetes and T2DM separately. However, there were only four studies [10, 11, 44, 45] in prediabetes. In consequence, we only examined the studies [12–14, 46–50] in T2DM. We did not detect any significant risk of publication bias in every outcome reported by those studies. The results of Egger’s regression test are summarized in Table 2. The funnel plots are illustrated in Supporting Information (S4 Fig).

**Table 2:** Egger’s regression test summary for publication bias of studies in type 2 diabetes mellitus.

Outcomes	Intercept	95% CI	p-value^a^
HbA1c [12–14,46,49,50]	-0.96	-5.72 to 3.80	0.604
FPG [12–14,46–50]	0.80	-2.84 to 4.45	0.608
TG [12–14,46–49]	-0.18	-9.14 to 8.78	0.960
TC [12–14,46–49]	1.83	-3.21 to 6.88	0.393
LDL [12–14,46,47,49]	2.91	-5.08 to 10.89	0.370
HDL [12–14,46,47,49]	-1.95	-17.20 to 13.29	0.740

CI, confidence interval; HbA1, glycosylated hemoglobin; FPG, fasting plasma glucose; TG, triglyceride; TC, total cholesterol; LDL, low density lipoprotein cholesterol; HDL, high density lipoprotein cholesterol

^a^Risk of publication is considered high if the intercept deviates significantly from zero with p-value <0.05.

## Discussion

The proposed mechanisms of curcumin antidiabetic effects were demonstrated through a whole picture of insulin resistance inhibition and some highlighted mechanisms. Curcumin improves insulin sensitivity by affecting three processes. Firstly, curcumin ameliorates glucose homeostasis by triggering glucokinase activity in the liver. Secondly, it induces lipid metabolism by raising lipoprotein lipase activity to reduce triglyceride. Thirdly, curcumin affects insulin pathway independently by inducing glucose transporter-4 (GLUT4) expression to increase peripheral glucose uptake. [51]. Additionally, curcumin attenuates tumor necrosis factor-alpha, plasma free fatty acid, and thiobarbituric acid reactive substances level as well as the activity of sorbitol dehydrogenase [52]. Interestingly, antihyperglycemic effect of curcumin and its analogues might be compared to the approved antidiabetic agent namely thiazolidinedione group. Curcumin activating PPAR-γ appears to offer good combination effect which improves insulin secretion, lipid metabolism, and free fatty acid receptor expression [8, 9]. Thus, all of these mechanisms may reflect glucose and lipid lowering effects in human.

The results of this investigation revealed the effect of curcumin on glycemic outcomes in both prediabetes and T2DM participants. The primary outcome on glycemic control in this research was HbA1c. We considered this outcome due to its representative measurement of long-term glycemic control in diabetes management. The trend of the glucose level is more reliably predicted by HbA1c than FPG which only demonstrates the blood glucose concentration at certain time. However, both HbA1c and FPG may be taken together since these parameters had a strong correlation [53]. Therefore, we set FPG as the secondary outcome. Assessment of 2-hours postprandial plasma glucose (2HPP) was supposed to be combined with those outcomes to achieve the target in management of both prediabetes and diabetes [54]. Despite this, we did not manage to perform meta-analysis on 2HPP. Respectively only one study in prediabetes [44] and the other in T2DM [47] provided this outcome data. Nevertheless, curcumin demonstrated meaningful effect on HbA1 reduction and tended to improve FPG in prediabetes. Furthermore, curcumin supplementation offered excellent effects on both HbA1c and FPG reductions in T2DM.

The effect of curcumin on glycemic level in both prediabetes and T2DM should reflect their corresponding influence on lipid profile. In fact, both glucose and lipid encounter such complex metabolism in the body. The abnormality of either glucose or lipid probably leads to a causal relationship [55]. Furthermore, glycemic control, particularly HbA1c, might estimate the presence of dyslipidemia in T2DM. This possible prediction is by the reason of the linear correlation between HbA1c and TC, TG, LDL, and HDL. Higher level of HbA1c tends to represent higher level of TC, TG, and LDL but lower level of HDL [56]. Lipid abnormality can be noticed not only in T2DM, but also in prediabetes. Again, this characterization might occur when HbA1c is involved in the prediction [57]. The results on lipid parameters in this study did not completely decline from this concept. Notwithstanding the non-statistically significant results on lipid parameters, the results were positive and consistent with those of glycemic parameters in both prediabetes and T2DM. Of these results on lipid outcomes, tendency of greater magnitude was seen in T2DM population. An important issue was bioavailabilty of curcumin. Several studies found that the levels of curcumin and its in vivo metabolites are low in serum and tissues [58–60].

We confirmed our findings in this meta-analysis by conducting sensitivity analysis. As we established strict criteria of treatment duration regarding appropriate period for HbA1c to be morethan 8 weeks, we found that most of the included studies were undertaken within eight weeks until three months. However, there were studies conducted much longer, respectively up to nine months in prediabetes [44] and six months in T2DM [14]. Therefore, we decided to exclude these studies in respective analyses to observe the estimated effects on both glycemic control and lipid outcomes in the majority of the studies length. The limited number of studies led us to perform the sensitivity analysis only in T2DM. Engaging with sample-size factor, there was likely small-trial effect of curcumin on glycemic control in T2DM. Some smaller individual studies [12,13,48,49] seemed to contribute for significant reduction in the whole meta-analysis together with the larger trial in longer duration [14]. However, when the larger trial was removed, we found that treatment with curcumin within 2 until 3 months might not be sufficient for glycemic control in T2DM. Meanwhile, the sensitivity analysis in lipid outcomes has confirmed the robustness pertaining that study duration did not affect changes on lipid profile.

Potential bias from the included studies might become another contributing factor for the results. Overall studies had low risk of bias, but half of studies unclearly described the concealment and assessment processes. Also, one study was not double-blinded. It should be recognized that trials conducted without adequate concealment and blinding might overestimate the treatment effects. Recent evidence proved that the average risk of bias of these sources probably exaggerated the results of trials, particularly greater in trials with subjective outcomes than trials with objective outcomes [61]. However, the present study assessed objective outcomes including laboratory-based values in both glycemic control and lipid profiles. Therefore, these issues should be negligible in general evaluation. Additionally, apparent publication bias of the included studies was not found in this study. Language of publication also seemed not to affect the publication bias since two of those studies were published in non-English language [12,50]. Thus, the minimized bias among the included trials should support the results in this study to establish the role of curcumin supplementation in clinical relevance.

This present systematic review and meta-analysis may strengthen the available evidences of curcumin becoming alternative adjunctive therapy to better control glycemic targets and lipid parameters. Some previous meta-analyses of RCTs of curcumin have been undertaken to assess the effects of curcumin on blood glucose and/ or lipid profile [62–66]. On the one hand, one meta-analysis has successfully demonstrated curcumin’s effective FPG reduction in dysglycemia comprising prediabetes, metabolic syndrome, and diabetic subjects [62]. Pure curcumin was proposed to affect more significantly both FPG and HbA1c reduction than turmeric preparation disregarding either in diabetic or non-diabetic subjects. Another meta-analysis has assessed not only glycemic parameters, but also lipid profile involving similar population with metabolic syndrome and related disorders [63]. Since this meta-analysis was published, we found 2 additional studies and therefore included in our meta-analysis. Concerningtheir several subgroup analyses [63], such as based on diseases (T2DM, obese and overweight) or short duration of treatment (included 4 weeks duration) curcumin was considered to affect glycemic parameters, lipid profile, and insulin resistance. The HbA1c test tells an average level of blood glucose over the past 2 to 3 months, therefore including more than 8 weeks duration was rather appropriate.

On the other hand, the results from the other three meta-analyses evaluating lipid outcomes were inconsistent. Two meta-analyses shared common evaluation approaches including varied population backgrounds and trial duration within seven days to six months [64,65]. However, only the larger study [65] has succeeded to present remarkable TG reduction and HDL elevation regardless of treatment duration. The third meta-analysis [66] analyzed the effect in population with high risk of cardiovascular diseases pooling metabolic syndrome and T2DM together. The results revealed significant decrease in LDL and TG. Subgroup analysis on TC convinced each particular benefit of turmeric extract and curcumin in metabolic syndrome. However, these significant results seemed to introduce bias due to some unexplained removals of study in the analysis.

Compared to previous studies, this current meta-analysis considers some more suitable approaches to investigate curcumin effects in specific population namely prediabetes and T2DM, respectively. For example, both glycemic and lipid outcomes were observed simultaneously; trial conducted for less than two months was not allowed; and more searches were conducted including non-English articles. Instead of performing sub-analyses with certain criteria under such broad population group of metabolic diseases, we defined strict criteria right at the beginning of the search. Hence, our systematic review and meta-analysis may grant more robust evidence to assist the application of curcumin supplementation in prediabetes and T2DM.

Our findings should be taken with caution. Heterogeneity should be considered and may be due to varied participants’ and studies’ characteristics. For example, studies’ duration, participants’ comorbidities, curcumin doses and preparations, co-medication, and lifestyle influence involved in each study might be influenced. However, looking further into individual studies suggested the following considerations. Firstly, under the same amount of administration, curcumin extract either pure curcumin or curcuminoids may be more beneficial than powdered turmeric to produce effects. This suggestion should concern that curcuminoids content in turmeric powder is only around 2–6% [67]. Thus, turmeric powder has very low dose of curcumin. Secondly, eight weeks seemed to be sufficient as minimum length of curcumin supplementation to start gaining benefit on glycemic control [11,12]. Meanwhile, duration longer than eight weeks may be required to obtain obvious results on lipid outcomes. Nonetheless, duration of curcumin treatment might require to follow the other contributing factors due to the finding of small-trial effect in our meta-analysis.

The other consideration concerning heterogeneity is co-medication during the treatment with curcumin. Co-medication may associate with the individual’s stage of the disease either prediabetes or diabetes. Our finding suggest that curcumin supplementation may be helpful in prediabetes without co-medication, but not in T2DM. However, the greater effects magnitude was mostly seen in T2DM than in prediabetic population. Thus, suggestion for taking curcumin in clinical practice should be concerned case by case following individual’s stage of disease. Also, the individual should be encouraged to keep maintaining healthy lifestyle while consuming curcumin. The data available draw mainly from Asian studies. This is because the majority of the studies included in this meta-analysis involved Asians.

Curcumin and its preparations demonstrated tolerable safety profile. Serious adverse events (AEs) were not found during the supplementation with curcumin, although some minor AEs were reported [10, 11, 14, 44–47]. A separate meta-analysis has been performed to confirm this safety consideration (S5 Fig). Curcumin might be related to rare AEs. However, the probability of curcumin-related AEs should not be ignored without attention. According to a computational study in regard to animal studies, prolonged consumption of curcumin was predicted to have tendency of dose-dependent hepatotoxicity in human [68]. Despite some included studies have reported insignificant harmful alteration in liver function [11, 13, 14, 44], clinical decision should be carefully concerned for long term curcumin administration in prone subjects. Safe dose of curcumin intake was mentioned up to 12 g/day as standardized curcuminoids extract in healthy people [69]. Nevertheless, based on the findings in this systematic review and meta-analysis, effective and safe administration of curcumin in prediabetes and T2DM are likely to be achieved with dose up to 1.8 g/day of curcuminoids extract and nine months of duration.

Some limitations in this systematic review and meta-analysis exist. We found one study [11] in prediabetes providing significantly different baseline in HbA1c and TG between the curcumin and placebo groups. This may introduce bias, although the pooled result was not dominated by this study. Next, more sample size might add more statistical power into the analysis. However, the available RCTs are lacking regarding curcumin’s effects on glycemic control and lipid profile in prediabetes and T2DM. Regardless of the small number of the included studies, heterogeneity could not be avoided. Also, studies which assessed pure curcumin are limited, so this meta-analysis still involved some differed preparations of curcumin. Taking all of these together, further and larger clinical trials evaluating the effects of curcumin or its specific dosage form on glycemic and lipid outcomes are expected, particularly in prediabetes and T2DM.

In conclusion, the findings of this systematic review may encourage supplementation of curcumin and its preparation specifically in Asian population with prediabetes and T2DM patient. Curcumin appears to offer meaningful effect on glycemic control, particularly HbA1c. Lack of effects in lipid outcomes were observed, but there was tendency of improvement in these outcomes with greater effect in T2DM. Curcumin and its preparation also demonstrate tolerable safety concern in the administration for eight weeks up to nine months. Hence, this evidence may uphold the role of curcumin including prevention and management in diabetes. Nevertheless, the application of curcumin supplementation in clinical practice should be taken with individual’s contributing factors.

## Supporting information

S1 Checklist PRISMA 2009 checklist. (DOC)

S1 Fig Risk of bias graph across all included studies. (TIF)

S2 Fig Forest plots of effects of curcumin compared to placebo on lipid outcomes in prediabetes. (DOCX)

S3 Fig Forest plots of effects of curcumin compared to placebo on lipid outcomes in type 2 diabetes mellitus. (DOCX)

S4 Fig Funnel plots of publication bias on glycemic and lipid outcomes in type 2 diabetes mellitus. Publication bias was assessed by Egger’s regression test and generated by StatDirect version 3. A, glycosylated hemoglobin; B, fasting plasma glucose; C, triglyceride; D, total cholesterol; E, LDL cholesterol; F, HDL cholesterol.
(DOCX)

S5 Fig Meta-analysis of adverse events in prediabetes and type 2 diabetes mellitus involving curcumin and placebo groups. (DOCX)

S1 Table Summary of sensitivity analysis in type 2 diabetes mellitus. HbA1c, glycosylated hemoglobin; FPG, fasting plasma glucose; TG, triglyceride; TC, total cholesterol; LDL, low-density lipoprotein; HDL, high-density lipoprotein; N, sample size; MD, mean difference.
(DOCX)
